# Clinical Characteristics and Early Interventional Responses in Patients with Severe COVID-19 Pneumonia

**DOI:** 10.1155/2021/6676987

**Published:** 2021-05-31

**Authors:** Susu He, Lina Fang, Lingzhen Xia, Shuangxiang Lin, Junhui Ye, Dinghai Luo

**Affiliations:** ^1^Department of Respiratory Medicine, Taizhou Hospital of Zhejiang Province Affiliated to Wenzhou Medical University, Linhai, Zhejiang, China; ^2^Endoscopy Center, Taizhou Hospital of Zhejiang Province Affiliated to Wenzhou Medical University, Linhai, Taizhou, China; ^3^General Practice, Taizhou Central Hospital, Taizhou, Zhejiang, China; ^4^Department of Radiology, Taizhou Hospital of Zhejiang Province Affiliated to Wenzhou Medical University, Linhai, Zhejiang, China; ^5^Department of Respiratory Medicine, The People's Hospital of Sanmen, Taizhou, Zhejiang, China; ^6^Department of Gastroenterology, Taizhou Hospital of Zhejiang Province Affiliated to Wenzhou Medical University, Linhai, Taizhou, China

## Abstract

Progressive acute respiratory distress syndrome (ARDS) is the most lethal cause in patients with severe COVID-19 pneumonia due to uncontrolled inflammatory reaction, for which we found that early intervention of combined treatment with methylprednisolone and human immunoglobulin is a highly effective therapy to improve the prognosis of COVID-19-induced pneumonia patients. *Objective*. Herein, we have demonstrated the clinical manifestations, laboratory, and radiological characteristics of patients with severe Coronavirus Disease-2019 (COVID-19) pneumonia, as well as measures to ensure early diagnosis and intervention for improving clinical outcomes of COVID-19 patients. *Summary Background Data*. The COVID-19 is a new infection caused by a severe acute respiratory syndrome- (SARS-) like coronavirus that emerged in China in December 2019 and has claimed millions of lives. *Methods*. We included 37 severe COVID-19 pneumonia patients who were hospitalized at Taizhou Public Health Medical Center in Zhejiang province from January 17, 2020, to February 18, 2020. Demographic, clinical, and laboratory features; imaging characteristics; treatment history; and clinical outcomes of all patients were collected from electronic medical records. *Results*. The patients' mean age was 54 years (interquartile range, 43−64), with a slightly higher male preponderance (57%). The most common clinical features of COVID-19 pneumonia were fever (29 (78%)), dry cough (28 (76%)), dyspnea (9 (24%)), and fatigue (9 (24%)). Serum interleukin (IL)-6 and IL-10 were elevated in 35 (95%) and 19 (51%) patients, respectively. Chest computerized tomography scan revealed bilateral pneumonia in 35 (95%) patients. Early intervention with a combination of methylprednisolone and human immunoglobulin was highly effective in improving the prognosis of these patients. *Conclusions*. Progressive acute respiratory distress syndrome is the most common cause of death in patients with severe COVID-19 pneumonia owing to an uncontrolled inflammatory response. Early intervention with methylprednisolone and human immunoglobulin was highly effective in improving their prognosis.

## 1. Introduction

In December 2019, a novel coronavirus was identified in patients with viral pneumonia in Wuhan, which was later named Coronavirus Disease-2019 (COVID-19) by the World Health Organization (WHO) on January 11, 2020 [1, 2]. Given the possibility of airborne transmission in humans, the virus has infected more than 100 million people and spread worldwide into hundreds of countries [3–5]. Most coronaviruses usually cause mild illness, but there are two *β*-coronaviruses, severe acute respiratory syndrome (SARS)-coronavirus and Middle-East respiratory syndrome (MERS)-coronavirus, which can lead to severe acute respiratory syndrome with a mortality rate of 10% and 37%, respectively [6, 7]. Recent studies have revealed that COVID-19 causes severe pneumonia, respiratory distress syndrome, and multiple organ failure, leading to a high mortality rate [8–10].

This study is aimed at describing the clinical, laboratory, and radiological characteristics of critically ill patients with COVID-19, as well as the effective outcomes after early detection and intervention. These findings could provide a useful medicinal strategy for the treatment of severely ill patients with COVID-19 pneumonia.

## 2. Materials and Methods

### 2.1. Ethics

This study was approved by the ethics committee of the Enze Hospital of the Zhejiang Enze Medical Center (group). Data collected from enrolled cases were shared with the WHO. Written informed consent was obtained from all patients before data collection.

### 2.2. Clinical Records and Data Collection

Thirty-seven adult patients with severe COVID-19 pneumonia, diagnosed following the WHO interim guidelines [1, 11], were hospitalized at Taizhou Public Health Medical Center in Taizhou City, Zhejiang Province from January 17, 2020, to March 11, 2020. The medical records obtained from patients were analyzed by the respiratory research team of Zhejiang Enze Medical Center (group) Taizhou Hospital and Enze Hospital. The clinical features; laboratory investigations; chest imaging characteristics; treatment history, including antiviral therapy, hormone therapy, human immunoglobulin therapy, and respiratory support; and recovery data were retrieved from electronic medical records. The source data included demographic data; symptoms; comorbidities; laboratory results; chest computerized tomography (CT) scan; and treatment measures, including laboratory results, such as complete blood count, blood clotting parameters, liver and kidney functions, serum electrolytes, erythrocyte sedimentation rate, C-reactive protein (CRP) level, procalcitonin (PCT) level, creatine kinase level, blood gas analysis, troponin level, and cytokine levels. All data were examined by two physicians.

### 2.3. Laboratory Investigations

Real-time fluorescent polymerase chain reaction (RT-PCR) was used to confirm novel coronavirus infection by detecting viral nuclei from respiratory tract specimens. Diagnosing severe respiratory symptoms requires fulfilling an oxygenation index criterion (PaO_2_/FIO_2_ of <300 mmHg). Clinical stability was defined as an oxygenation index of ≥300 mmHg with stable clinical symptoms. The time of symptom remission was defined as the time from the diagnosis of severe illness to the time of symptom relief. The time of oxygenation improvement was the time of diagnosis of severe disease to the time of oxygenation index of ≥300 mmHg. The apparent absorption time of the internal lesion was regarded as the time from the diagnosis of severe disease till obvious absorption of the pulmonary lesion on CT. The discharge criteria were defined as normal body temperature for more >3 days, significant improvement of respiratory symptoms, pulmonary imaging showing significant inflammatory absorption, and two consecutive negative respiratory nucleic acid test results (sampling interval of at least >24 h).

### 2.4. Medical Treatment

Laboratory tests and chest CT were performed on the patients on admission. Next, 5 million units of aerosolized *α*-interferon in combination with oral lopinavir/ritonavir (500 mg) were administered twice daily to reduce viral activity. During hospitalization, vital signs and blood oxygen saturation were closely monitored. Blood gas analysis was performed promptly to determine the oxygenation index and the development of severe or new symptoms (chest tightness) were monitored. Respiratory support (high flow oxygen inhalation through a nasal catheter) was immediately administered to severely ill patients along with intravenous methylprednisolone (0.5 − 1 mg/kg daily), human immunoglobulin (0.3 − 0.5 g/kg daily), and fluids. Albendazole tablets (200 mg thrice daily) were administered to increase the efficacy of antiviral drugs. Human immunoglobulin was stopped based on the patients' condition, and the dose of methylprednisolone was gradually reduced accordingly. Empirical antibiotics were administered to patients who showed elevated white blood cell count and/or significantly elevated C-reactive protein (CRP) level. Critically ill patients were evaluated for oxygenation index at least once daily until clinical signs and symptoms were relieved.

### 2.5. Statistical Analyses

The categorical variables were described as frequency and percentages, and the continuous variables were described using mean, median, and interquartile range (IQR). All statistical analyses were performed using SPSS (version 20.0) software (IBM, Armonk, NY, USA).

## 3. Results

The study population consisted of 37 critically ill inpatients diagnosed with COVID-19 pneumonia. The mean age of the patients with severe COVID-19 pneumonia was 54 years (IQR, 43−64), with a slightly higher male preponderance (57%). Nine (24%) patients had one or more comorbidities. The most common clinical features of COVID-19 pneumonia were fever (29 (78%)), dry cough (28 (76%)), dyspnea (9 (24%)), and fatigue (9 (24%)). As of March 11, 2020, all patients were discharged (Table 1).

At admission, patients had absolute lymphocytosis (28 (76%)) and thrombocytopenia (7 (19%)), but leukopenia was rare (2 (5%)). Among the coagulation parameters, only one (3%) patient showed a slightly increased activated partial prothrombin time, two (5%) showed a decreased prothrombin time, 28 (76%) showed a decreased D-dimer level, and a few (9 (24%)) showed an increased D-dimer level (IQR, 0.22−0.71 *μ*g/mL). Liver function was impaired to varying degrees in nine (24%) patients with elevated alanine aminotransferase/aspartate aminotransferase levels, and renal function was impaired in five (14%) patients with elevated creatinine levels. A slightly increased creatine kinase level was found in eight (22%) patients. The troponin levels were in the normal range in all patients.

A vast majority of patients (32 [86%]) showed an increased CRP level (IQR, 10.0–50.8 mg/L). Thirty-one (84%) patients had an increased erythrocyte sedimentation rate (IQR, 29.5–54.5 mm/h). Serum PCT levels were partially increased in 14 (38%) patients, although it was not significant (IQR, 0.03−0.07 ng/mL). Serum interleukin (IL)-6 and IL-10 levels were elevated in 35 (95%) and 19 (51%) patients, respectively (Table 2).

Abnormal CT findings were detected in all patients. Only two (5%) patients had unilateral lobar lesions, while the remaining 35 (95%) had bilateral lobar lesions. Chest CT in most patients showed multiple manifestations, the most common being a patch shadow, which was found in all patients. The other findings were ground glass shadows (27 (73%)), interstitial changes (25 (68%)), consolidation shadows (22 (59%)), and nodular shadows without pleural effusion (10 (27%)) (Table 3).

All patients received oxygen; 32 (86%) and five (14%) patients received high-flow oxygen through a nasal catheter without invasive ventilation. All patients were treated with 5 million units of aerosolized *α*-interferon and lopinavir/ritonavir therapy (500 mg, twice daily). Albendazole tablets (200 mg thrice daily) were administered to 23 (62%) patients. Based on the white blood cell count and CRP level, nine (24%) patients were treated with antibiotics, including penicillin, macrocyclic lipids, and quinolones. The duration of antibiotic treatment was 2–11 days (median, 7 days; IQR, 4.5–7.4). Thirty (81%) patients received intravenous methylprednisolone intravenous infusion (0.5−1 mg/kg daily) for was 3−18 days (median, 7 days; IQR, 4−11 days), depending on the clinical condition. Twenty-five (68%) patients were treated with human immunoglobulin (0.3–0.5 g/kg daily), and 24 (65%) of them were treated for 3–11 days (median, 4 days; IQR, 3–5.5) (Table 4).

The median duration from symptom onset to diagnosis of severe illness was 7.5 days (IQR, 4.5–7.5), the median duration for symptom remission was 5 days (IQR, 2.5–11), and the median duration for saturation improvement was 5 days (IQR, 3–9). Significant absorption of pulmonary lesions was observed in 28 (76%) patients within a median duration of 9 days (IQR, 6–11) (Table 5).

## 4. Discussion

Among the 37 laboratory-confirmed severe COVID-19 patients, nine (24%) had underlying diseases, mainly hypertension, but a significant number of previously healthy patients had worsened clinical status during treatment. The main symptoms of patients with severe infection are fever, dry cough, chest tightness, and weakness. A few patients may have muscle pain, pharyngeal pain, dizziness, headache, loss of appetite, etc. COVID-19 patients rarely have gastrointestinal symptoms, such as diarrhea, which is different from the symptoms of SARS-coronavirus and MERS-coronavirus infections [11, 12].

Similar to recent reports [13–15], a reduced absolute lymphocyte count was found in 76% of critically ill patients. Reduced IL-6 and IL-10 levels were found in 95% and 19% of patients, respectively, suggesting that COVID-19 may have a role in cellular immune deficiency. The virus spreads through the mucous membrane along the respiratory tract, which provokes a series of immune reactions leading to cytokine storm, eventually causing a change in the peripheral blood lymphocyte count. IL-6 may play a proinflammatory role in pulmonary inflammation, and a significant increase in IL-6 level was found in the majority of patients, suggesting that severe COVID-19 may cause a significant exudation of IL-6 into the lungs. A decrease in the absolute lymphocyte count and increased IL-6 and IL-10 levels may indicate disease worsening.

In our study, PCT level, D-dimer level, clotting parameters, and troponin level were not much altered or slightly elevated, unlike in previous reports involving patients infected with SARS-CoV and MERS-CoV [16]. We speculate that our patients were not critically ill enough to require intensive care and did not develop coagulation disorders, liver and kidney dysfunctions, and myocardial injuries. Furthermore, it also suggests that PCT level, coagulation parameters, troponin level, and other common indicators cannot predict disease worsening.

Chest CT of patients with severe COVID-19 mainly shows bilateral patchy and frosted glass shadows. In our study, the involvement of multiple lobes was found in most patients, some of them showed consolidations, interstitial changes, and nodule shadows. No patient showed pleural effusion. The oxygenation index is a sensitive indicator of the progress of COVID-19. Patients diagnosed with COVID-19 were closely monitored for vital signs immediately after admission, and oxygen saturation was measured twice daily. Blood gas analysis was also performed periodically.

We evaluated the pattern of changes in symptoms. Disease aggravation was reflected by chest tightness. To detect disease progression early, blood gas analysis should be performed immediately to determine the oxygenation index. Because some patients cannot withstand imaging due to advanced disease, and imaging findings may be detected much late (advanced disease), it is not recommended to intervene after the appearance of chest CT features [17, 18].

In patients diagnosed with COVID-19, we immediately administered *α*-interferon along with lopinavir/ritonavir. However, a considerable number of patients were in the critical stage, suggesting that the antiviral drugs may not be as efficacious as expected. Many patients had diarrhea and other adverse effects; hence, the administration of antiviral drugs remains to be discussed further.

For the diagnosis of severe COVID-19, inflammatory mediators produced by viral infections need to be assessed [19, 20]. Considering cytokine storm, short-term use of a small dose of corticosteroid can reduce the risk of acute respiratory distress syndrome [21]. Therefore, methylprednisolone (0.5−1 mg/kg) was administered to most patients in addition to human immunoglobulin in order to prevent cytokine storm. After patients showed a good response, the oxygenation index returned to ≥300 mmHg. The intervention continued for an average of 9 days after review. Timely administration of glucocorticoids and human immunoglobulin could effectively inhibit the progression of COVID-19 and reverse the condition [22, 23]. However, it needs further study whether glucocorticoids prolong the time of virus excretion from the body. In the treatment of severely ill COVID-19 patients, we added albendazole, whose efficacy against COVID-19 needs further evaluation.

Severe COVID-19 patients were subjected to early intervention under close monitoring. All patients improved and could be discharged alive, which is notably different from previous reports [21, 24]. We believe that the severity of the disease is independent of its prognosis [25, 26], suggesting that symptoms, clinical signs, laboratory results, and chest imaging findings are more reliable for assessing the prognosis of COVID-19 pneumonia.

Progressive acute respiratory distress syndrome is the most common cause of death in patients with severe COVID-19 pneumonia owing to an uncontrolled inflammatory response. Early isolation, early diagnosis, and early treatment with methylprednisolone and human immunoglobulin can reduce the mortality rate of patients with COVID-19 pneumonia.

## Figures and Tables

**Table 1:** Baseline characteristics of patients infected with COVID-19. Data are median (IQR) or *n*/*N* (%), where *N* is the total number of patients with available data.

Patients (*n* = 37)	
Age, years	
Median (IQR)	54 (43-64)
Range	27-86
<40	6 (16%)
40-70	30 (81%)
>70	1 (3%)
Sex	
Male	21 (57%)
Female	16 (43%)
Current smoking	3 (8%)
Comorbidity	9 (24%)
Hypertension	6 (16%)
Diabetes	2 (5%)
Chronic obstructive pulmonary disease	2 (5%)
Hypothyroidism	2 (5%)
Signs and symptoms at admission	
Fever	29 (78%)
Cough	28 (76%)
Sputum production	6 (16%)
Dyspnea	9 (24%)
Myalgia	3 (8%)
Fatigue	8 (22%)
Diarrhea	3 (8%)
Headache	4 (11%)
Dizzy	5 (14%)
Pharyngula	3 (8%)
More than one sign or symptom	32 (86%)
Clinical outcome	
Discharged	37 (100%)
Died	0 (0%)

**Table 2:** Laboratory findings of patients infected with COVID-19.

Blood routine	Patients (*n* = 37)
Leucocytes (×109 per L; normal range 3.5–9.5)	6 (4.3-7.6)
Increased	5 (14%)
Decreased	2 (5%)
Neutrophils (×109 per L; normal range 1.8–6.3)	4.5 (2.7-6.6)
Increased	9 (24%)
Lymphocytes (×109 per L; normal range 1.1–3.2)	0.8 (0.6-1.0)
Decreased	28 (76%)
Platelets (×109 per L; normal range 125.0–350.0)	200 (141-258)
Increased	1 (3%)
Decreased	7 (19%)
Coagulation function	
Activated partial thromboplastin time (normal range 23.5–36.0)	30.2 (28.1-32.7)
Increased	1 (3%)
Decreased	0 (0%)
Prothrombin time (s; normal range 12.5–14.0)	11.9 (11.3-12.5)
Increased	2 (5%)
Decreased	28 (76%)
D-dimer (*μ*g/L; normal range 0.0–0.55)	0.32 (0.22-0.71)
Increased	9 (24%)
Blood biochemistry	
Alanine aminotransferase (U/L; normal range 9.0–50.0) ALT	22 (16.5-36)
Increased	7 (19%)
Aspartate aminotransferase (U/L; normal range 15.0–40.0) AST	28 (21.5-39.5)
Increased	9 (24%)
Serum creatinine (*μ*mol/L; normal range 62.0–97.0)	42 (29.5-54.5)
Increased	5 (14%)
Creatine kinase (U/L; normal range 38.0–174.0)	88 (66.5-161.5)
Increased	8 (22%)
Troponin(ng/mL; normal range 0.00-0.08)	0.01 (0.01)
Increased	0 (0%)
Infection-related biomarkers	
C-reactive protein (mg/L; normal range 0.0–5.0)	19.1 (10.0-50.8)
Increased	32 (86%)
Erythrocyte sedimentation rate (mm/h; normal range 0.0–20.0)	42 (29.5-54.5)
Increased	31 (84%)
Procalcitonin (ng/mL; normal range 0.0–0.05)	0.05 (0.03-0.07)
Increased	14 (38%)
Interleukin-6 (pg/mL; normal range 0.1–2.9)	12.85 (6.3-27.7)
Increased	35 (95%)
Interleukin-10 (pg/mL; normal range 0.1–5.0)	5.1 (3.4-9.2)
Increased	19 (51%)

**Table 3:** Radiographic findings of patients infected with COVID-19.

Patients (*n* = 37)	
Ground-glass opacity	27 (73%)
Patch shadow	37 (100%)
Interstitial abnormalities	25 (68%)
Consolidation	22 (59%)
Nodule	10 (27%)
Normal	0 (0%)
Local patchy shadowing	2 (5%)
Bilateral patchy shadowing	35 (95%)

Data are *n*/*N* (%), where *N* is the total number of patients with available data.

**Table 4:** Treatment of patients infected with COVID-19.

	*n*/*N* (%)	Median (IQR)
No. of patients	37	37
Oxygen therapy		
Nasal cannula	32 (86%)	NA
High-flow nasal cannula	5 (14%)	NA
Antiviral treatment		NA
*α*-Interferon	37 (100%)	NA
Lopinavir/litonavir	37 (100%)	NA
Arbidol	23 (62%)	NA
Glucocorticoids	30 (81%)	7 (4-11)
Intravenous immunoglobulin therapy	25 (68%)	4 (3-5.5)
Antibiotic treatment	9 (24%)	7 (4.5-7.5)

Data are median (IQR) or *n*/*N* (%), where *N* is the total number of patients with available data.

**Table 5:** Clinical outcome of patients infected with COVID-19.

	Patients, *n*	Median (IQR), days
Time of severe	37	7.5 (4.5-7.5)
Time of symptom remission	37	5 (3-10)
The time of oxygenation improvement	37	5 (3-9)
Obvious absorption time of intrapulmonary lesion	28	9 (6-11)

Data are median (IQR). Time of severe was onset of symptoms to the diagnosis of severe, symptoms diagnosed with severe time represent the time to relieve symptoms, improve oxygenation time expressed as a diagnosis of severe oxygenation index of 300 mmHg or to time, and lung lesions significantly absorbed within the said time view demonstrate the focal area of the lungs to the CT diagnosis of severe time, one of the most obvious time to absorb the time obviously. One patient is still in a critical stage.

## Data Availability

The data included in this paper are available without any restriction.
